The article "Design of Structural Parameters of Cutters for Tea Harvest Based on Biomimetic Methodology" was published in 2021. Journal: Appl Bionics Biomech.

# Design of Structural Parameters of Cutters for Tea Harvest Based on Biomimetic Methodology

**DOI:** 10.1155/2021/8798299

**Published:** 2021-07-22

**Authors:** Zhe Du, Yongguang Hu, Yongzong Lu, Jing Pang, Xinping Li

**Affiliations:** ^1^College of Agricultural Equipment Engineering, Henan University of Science and Technology, Luoyang 471023, China; ^2^School of Agricultural Engineering, Institute of Agricultural Engineering, Jiangsu University, Zhenjiang 212013, China

## Abstract

Owing to their sharp teeth, crickets can eat through new shoots of the stalks of tea plants. Inspired by the special geometrical structure of the teeth of crickets, this study designed a biomimetic cutter to reduce the force and energy required to cut the stalks of tea plants. Therefore, four biomimetic cutters were considered: *a*, *b*, *c*, and *d*. Cutter *a* was a traditional cutter used for comparison with the other three cutters, which were biomimetic. The cutters were manufactured using 3D printing technology and assessed by a texture tester at different loading speeds (5, 10, and 15 mm/s, respectively). The results show that cutter *c* delivered better performance compared to cutter *a* at loading speeds of 5, 10, and 15 mm/s, respectively. However, at 15 mm/s loading speed, the maximum cutting forces required for cutters *b* and *c* were 9.43% and 6.04% lower, respectively, than that for cutter *a* (9.021 N). Similarly, the energies consumed by cutters *b* and *c* were 13.8% and 4.24% lower than that consumed by cutter *a* (1.225 J). In addition, cutter *c* delivered the best results compared to others. Based on the study results, it was concluded that the biomimetic cutters can thus help to optimize the tea harvest.

## 1. Introduction

Tea is an aromatic beverage that is consumed all over the world [1]. Tea pluckers are widely used to improve the yield of harvesting tea plants [2, 3]. The cutter is a key component of the tea plucker that has a significant influence on its cutting performance and efficiency [4, 5]. Commonly used cutters in tea pluckers include the reciprocating cutter, disk cutter, and flail-type cutter. Compared with the disk and flail-type cutters, the reciprocating cutter has a simpler structure and a wider range of adaptations [6–8]. Besides, it is important to optimize the structural parameters of the reciprocating cutter to improve its cutting performance.

Present research on the optimal design of the reciprocating cutter has focused on its cutting speed, cutting angle, geometry, and size. The mechanical properties of the plant have also been considered in the design of the cutter [9–12]. To design a harvesting element, a study by Sunil et al. studied the mechanical properties of energycane stalks and found that the oblique angle and cutting speed of the cutter had a significant effect on the cutting energy [13]. Yamasaki et al. [14] and Galedar et al. [15] performed similar research on the structural parameters of the reciprocating cutter. Shi et al. [16] established the 3D models of crop stalks and cutters by using response surface methodology to determine the optimal combination of the kinematic parameters of the cutter at a cutting speed of 1.6 m/s, cutting angle of 15°, and working speed of 1 m/s.

The article "Design of Structural Parameters of Cutters for Tea Harvest Based on Biomimetic Methodology" was published in 2021. Journal: Appl Bionics Biomech.

Biomimetic technology has recently been applied to optimize the design of traditional agricultural machinery and to improve its energy utilization [17–20]. It combines biological principles with engineering problems for developing solutions. A study by Chang et al. [21] designed a biomimetic stubble cutter by imitating the outer contour of the foreclaws of the nymph of the species *Cryptotympana atrata* for reducing the cutting resistance. By considering the serrated incisors of a grasshopper, Jia et al. [22] designed and manufactured a biomimetic cutter to reduce the requirement of the maximum cutting force and cutting energy. Tong et al. [23] optimized a stubble-cutting disk based on the dynamics of the clawed toes of a mole rat as it digs the ground. Research in bionics can be consulted to design a cutter that can reduce the energy and the cutting force needed for harvesting [24, 25].

Biomimetic cutting techniques are usually based on the characteristics of phytophagous insects, such as the tiger beetle [26], bamboo weevil larva [27], and locust [28]. These insects have well-formed, strong mandibles to efficiently chew plants. Features of parts of their mouth can be used to optimize the parameters of a cutter. For the aggression of the mouth structure to be adaptive, insects must decide what angle is best to eat. How it is done is arguably best understood in crickets (Orthoptera: Gryllidae) [29]. The cricket is an omnivorous insect that consumes the fresh shoots, stalks, leaves, and seeds of tea plants, vegetables, and other crops. The teeth in its mandible have evolved and adapted so that they can easily cut into and tear plant fibers [30]. Therefore, features of the teeth of the mandible of the cricket can be used to design an efficient cutter for tea plants.

Based on the above discussion, the present paper examines the structural parameters of cutters for harvesting tea plants based on biomimetic technology. The line of the outer contour of the serrated structure on the mandible of the cricket is extracted, and its fitted curve was applied to design a biomimetic cutter. In addition, four cutters (*a*, *b*, *c*, and *d*) were manufactured by using 3D printing technology, and experiments were carried out on a texture tester to investigate their performance in terms of the required cutting force and energy. Finally, the cross-section of the tea stalk was observed by using a microcomputed tomography (micro-CT) scanner to analyze the performance of the cutters.

The article "Design of Structural Parameters of Cutters for Tea Harvest Based on Biomimetic Methodology" was published in 2021. Journal: Appl Bionics Biomech.

## 2. Materials and Methods

### 2.1. Cutter Design

#### 2.1.1. Sample Preparation

For the present experiment, the adult crickets were collected from the suburbs of Ningyang city in Shandong Province, China. Five samples were narcotized by 99% ether, and their teeth were taken out using tweezers and washed with distilled water. However, the tea samples were obtained from the Maichun Tea Farm in Danyang, Jiangsu, near the Yangtze River region (latitude 32°02′N, longitude 119°67′E). The experiment selected verity tea, and the tea stalk was the third internode of the Zhongcha 108 variety. At the time of the sampling, the average moisture content of the tea stalk was 73.8% (wet basis), and the picking time was June 2019 [31].

#### 2.1.2. Sample Observation

The geometric structure of the teeth of the crickets and the microstructure of the tea stalk were observed by a digital microsystem (VHX-900F, KEYENCE, Japan). This system was used to measure the 2D size and 3D outline of these objects. A photograph of the teeth on the mandible of the cricket is shown in Figure 1(a), and the structure of the tea stalk is shown in Figure 1(b).

#### 2.1.3. Curve Extraction

TRACE software was used to convert the bitmap into a vector graph for extracting the contours of the geometrical features of the teeth of the cricket. To easily separate the object from the background of the image, the vector graph was subjected to a binary process and was converted into a black-and-white image. Also, AutoCAD software was used to adjust and plot the points to extract the contour line of the serrated structure on the mandible of the cricket. The curve of the outer margin of the serrated structure was divided into individual curves to precisely express them at a given time. Finally, Origin software was used for data analysis to select the biomimetic units.

#### 2.1.4. Cutter Manufacture

The contours of the geometrical features of the teeth of the cricket were used in the design of biomimetic cutters. To accurately express the biomimetic element, 3D printing was used to machine the cutter by using Future 8000 resin. It has a highly precise and smooth surface and delivers a similar mechanical performance to that of acrylonitrile butadiene styrene (ABS). The 3D printed cutters were used in all tests. Besides, the cutter material was still Future 8000 resin in the simulation test.

The article "Design of Structural Parameters of Cutters for Tea Harvest Based on Biomimetic Methodology" was published in 2021. Journal: Appl Bionics Biomech.

### 2.2. Test Methods

The cutters used in the experiments were 1.5~2.5 mm thick. Finite element analysis using ANSYS software was carried out to determine the influence of the cutter thickness on the cutting force.

A texture tester (Stable Micro Systems, TA-XT2i) was used to measure, record, and analyze the cutting performance (cutting force and time and energy consumed) of different cutters on a tea stalk [32]. The tester had a wide range of moving distances of 0.1 mm–295 mm, and its accuracy of force measurement was 0.025% at a speed of 0.1~20 mm/s. The loading speed is an important factor because the tea stalk was made of viscoelastic material [33]. In the cutting experiments, the loading speeds were set to 5, 10, and 15 mm/s, respectively. When the cutter was cutting the tea stalk at a constant speed, the cutting force-displacement curve could be obtained with the texture tester. The energy consumed could be calculated by the area between the cutting curve and the displacement axis [22].

When the loading speed was 10 mm/s with a cutting force of 2.5 N, the cross-section of the tea stalk was changed. Moreover, X-ray microcomputed tomography (Scanco Medical AG, micro-CT 100, Switzerland) was used to scan the tested stalks after the cutting experiment. The X-ray tube had a spot size of 5 mm with an operating voltage of 45 kV and a current of 88 *μ*A. A total of 200 sliced images (each with 1024 × 1024 pixels) were obtained from the experiment. The tea stalk was fixed on a sponge in the scanning barrel to observe its internal structure.

## 3. Results and Discussion

### 3.1. Curve of the Tooth Structure

The teeth on the mandible of the cricket varied in terms of size and shape. Different arc-shaped structures of the teeth significantly reduced the frictional resistance between the mandible and the new shoots of the plant.

#### 3.1.1. Fitting Curve of the Serrated Structure

The arc-shaped structure of the teeth on the mandible of the cricket was divided into five curves (curves *a*–*e*). A nonlinear regression model was used to analyze the outer margin of curves *a* to *e*. The fitting of the curve of the serrated structure is given in the following equation:

(1) $$\begin{array}{c} y\left(x\right)=a_{0}+a_{1}x+a_{2}x^{2}+a_{3}x^{3}+a_{4}x^{4}. \end{array}$$

The fitting parameters of the tooth curve are presented in Table 1. It was found that the values of *R*^2^ for all curves (*a*, *b*, *c*, *d*, and *e*) were greater than 0.9595. Therefore, the results of fitting were acceptable.  Figure 2 shows curves *a*–*e*. Curves *a*, *c*, and *e* had the same trend of rise and fall, whereas curves *b* and *d* had slightly different ones. Curve *a* increased almost linearly while curves *c* and *e* were convex in their rising parts before decreasing. The peak value of curve *a* was larger than those of the other curves.

The article "Design of Structural Parameters of Cutters for Tea Harvest Based on Biomimetic Methodology" was published in 2021. Journal: Appl Bionics Biomech.

#### 3.1.2. Best Approximation of the Fitting Curve

The first sharp tooth (Figure 1(a)) on the mandible of the cricket cuts off the shoots efficiently, and the other teeth are used to grind the food [30, 34]. The first sharp tooth can reduce the cutting resistance as well. Curve *a*, which models this tooth, was thus selected to design the model of the cutter.

To reduce the difficulty of processing the cutter, curve *a* was replaced by the fitted curve and straight lines to simplify the shape of the tooth while retaining its bionic characteristics. In the fitted curve (and straight line), the sum of squares of the error was used as the optimum index to seek the best-matching function. When the fitted curve was used, the expression of curve *a* was a five-order polynomial equation with an *R*^2^ value of 0.999 (Figure 3). The fitting of the curve is presented in the following equation:

(2) $$\begin{array}{c} y\left(x\right)=0.16166+2.61437x+0.0356x^{2}-0.00562x^{3}-2.61\times 10^{-6}x^{4}+2.02\times 10^{-6}x^{5}. \end{array}$$

When the fitted straight line was used, curve *a* was fitted by the least squares method. The fitting function was set as in the following equation:

(3) $$\begin{array}{c} S\left(x\right)=b_{0}+b_{1}x. \end{array}$$

The least squares method was used for the rising and falling parts of the curve (Figure 4). The fitting parameters *b*_0_ and *b*_1_ were calculated using Origin software, as shown in Table 2. The slopes of the rising and falling parts on the approximate line segment were 1.959 and –1.891, respectively. In the Cartesian coordinate system, the corresponding dip angles were 63° and 118°, with corresponding *R*^2^ values of 0.964 and 0.953. These results indicated a high correlation between the fitted line and the true curve.

Therefore, the fitting curve and straight lines could replace the curve of the profile of the first tooth on the mandible of the cricket for simplifying the processing technology and retaining bionic characteristics.

#### 3.1.3. Cutter Design and Manufacture

Different cutters with no burrs on the corners are shown in Figure 5. Cutter *a* was a traditional cutter used for a comparison of cutting performance with the other cutters—*b*, *c*, and *d*—which were biomimetic. They were designed based on the curve of the structure of the first sharp tooth on the mandible of the cricket (i.e., curve *a*). The contour line of cutter *a* was trapezoidal. Those of cutters *b* and *c* were the fitted curve of Equation (2) and the fitted scalene triangle of Equation (3), respectively. The contour line of cutter *d* was a combination of a trapezoid and a scalene triangle. For cutters *c* and *d*, the angles of the two sides of the triangle along the vertical direction were 27° and 28°, respectively (Figure 6).

The article "Design of Structural Parameters of Cutters for Tea Harvest Based on Biomimetic Methodology" was published in 2021. Journal: Appl Bionics Biomech.

### 3.2. Analysis of the Cutter Thickness

Stress and deformation had a significant influence on the stability and wear of the cutter. Many factors in turn affect the stress and deformation of the cutter, such as its mechanical properties, type of cutter, and structural and motion-related parameters. The authors here examined the influence of the thickness of the cutter on the stress on it and its deformation.

Assuming that the load was 3 N, the finite element analysis showed that the stress field and deformation of the cutter changed with its thickness, as shown in Figure 7. The maximum equivalent stress of the cutter decreased first and then changed a little with increasing thickness. At different thicknesses of the cutter, the maximum equivalent stresses produced by cutters *b* and *c* were similar and lower than those produced by cutters *a* and *d*. With an increase in the cutter thickness, its total deformation decreased gradually. The trend of change in cutter *a* was prominent, whereas those of cutters *b*, *c*, and *d* went smoothly. When the thickness of the cutter was 1.5~2.5 mm, the maximum equivalent stress and total deformation produced by cutters *b* and *c* did not change significantly with thickness.

### 3.3. Experiment to Test Cutting Performance

#### 3.3.1. Cutting Force

The cutting force reflects the efficiency of cutting. To clearly examine the efficiency of the cutter, the maximum cutting force at loading speeds of 5, 10, and 15 mm/s was used (Table 3). The average maximum cutting force is shown in Figure 8.

At a loading speed of 5 mm/s, the average maximum forces of cutters *a*, *b*, *c*, and *d* were 9.086 N, 10.047 N, 8.987 N, and 9.195 N, respectively (Table 3 and Figure 8). The average maximum cutting forces of cutters *b* and *d* increased by 10.58% and 1.2%, respectively, compared with that of cutter *a*. However, the average maximum cutting force of cutter *c* was smaller than that of cutter *a* by 1.08%. The average maximum cutting forces of cutters *b*, *c*, and *d* were 9.193 N, 9.027 N, and 10.939 N, respectively, at a loading speed of 10 mm/s, smaller by 1.35% and 3.13% and larger by 17.4%, respectively, than that of cutter *a* (9.318 N). The average maximum cutting forces of cutters *a*, *b*, *c*, and *d* were 9.021 N, 8.171 N, 8.476 N, and 13.597 N, respectively, when the loading speed was 15 mm/s. In comparison with the average maximum cutting force of cutter *a*, those of cutters *b* and *c* were smaller by 9.43% and 6.04%, respectively, whereas that of cutter *d* was larger by 50.72%. With the increase in loading speed, the average maximum cutting forces of cutters *a*, *b*, and *c* showed no significant changes while that of cutter *d* increased.

The article "Design of Structural Parameters of Cutters for Tea Harvest Based on Biomimetic Methodology" was published in 2021. Journal: Appl Bionics Biomech.

The maximum cutting force used for the tea stalk was much higher than the general picking force of 2.59 N [35] because the cutters were made of Future 8000 resin, not steel. This also affected the time and energy needed for cutting. The cutting time and energy consumption are closely related to the structural parameters of the cutter. Because of differences in cutter shapes, the tea stalk was squeezed to varying degrees, and the cutting times and energies consumed by different cutters were different.

#### 3.3.2. Energy Consumption

Energy consumption is an important factor that reflects the efficiency of cutting. It can be represented by the area between the curve of the cutting force and the displacement axis [21]. When the loading speeds were 5, 10, and 15 mm/s, the energy consumed by the different cutters is recorded in Table 4 and their average energy consumption is shown in Figure 9.

At loading speeds of 5 and 10 mm/s, the average energy consumption of cutter *d* was higher than those of the other cutters (Table 4 and Figure 9). The average maximum cutting forces of cutters *a*, *b*, and *c* were similar. When the loading speed was 15 mm/s, the average energies consumed by cutters *a*, *b*, *c*, and *d* were 1.225 J, 1.056 J, 1.173 J, and 2.567 J, respectively. Compared with cutter *a*, the average maximum cutting forces of cutters *b* and *c* were smaller by 13.8% and 4.24%, respectively, whereas that of cutter *d* was larger by 109.55%.

The energy consumed by the biomimetic cutters *b* and *c* were lower than those consumed by the traditional cutter *a* and the biomimetic cutter *d*.

## 4. Discussion

### 4.1. Behavior Mechanism of Crickets

The studies had shown that insects could decide which angle to eat and when best to fight by the powers of neuromodulation [29]. With the genetic techniques, the neuron which influenced aggression had been found in the fruit fly. In crickets, though, we knew nothing about the neuron of the eat and fight. In addition, there were few studies on the effects of left-right asymmetries in the brain and behavior on crickets (invertebrates) when eating and fighting [36]. Therefore, further research is needed on the working mechanisms allowing left-right mandible bite behavior in crickets. This might be due to the difference in nervous innervation. Now that the genetic techniques are becoming available for crickets [37], it could be expected that more advances will occur in the future studies of the model system of crickets.

The article "Design of Structural Parameters of Cutters for Tea Harvest Based on Biomimetic Methodology" was published in 2021. Journal: Appl Bionics Biomech.

### 4.2. Cutting Mechanism of the Stalk

Images of structural changes to the tea stalk were observed using a micro-CT scanner and are shown in Figure 10. According to Figures 2 and 9, the structure of the tea stalk can be divided into four parts: the pith, xylem, phloem, and epidermis. A similar tissue structure was obtained by Li and Lai, who observed the microstructure of the tea stalk using a scanning electron microscope [38]. Within the structure of the tea stalk, the cutting force and energy needed for the pith were low. Hence, it was ignored owing to the heterogeneous nature of the tea stalk and its softer, spongy internal structure.

In Figures 10(b) and 10(c), the compressive deformation in the tea stalk before damage is shown. The xylem structure was damaged in the compression stage. The process of cutting the tea stalk can be divided into two stages. In the first stage, the cutting force was applied to the xylem, which is the tissue supporting the plant. The second stage involved the application of the cutting force to the epidermis and phloem, which are the mechanical tissues of the tea stalk. The epidermis and xylem caused the two peaks to appear in the curve of the cutting force (Figure 11). In Figure 11, the first and second peak values are the maximum forces that broke the xylem as well as the epidermis and phloem. A similar conclusion was obtained by Leblicq et al., who studied the deformation of the plant stalk as well as the interaction between the plant and the force. They found that the breaking of the stalk can be analyzed in two consecutive phases (ovalization and buckling) [39].

### 4.3. Comparative Analysis of the Cutter

In general, shearing is the most effective method to cut lignocellulose materials, such as tea stalks. When the tea stalk was cut using cutters *a*, *b*, and *c*, the contact surface of the cutters with the epidermis of the tea stalk formed a line. This style of contact is good for shearing. Cutters *b* and *c* required smaller cutting forces and energies than cutter *a*, which indicates that they can better cut lignocellulose materials. This is because cutters *b* and *c* are biomimetic cutters with a special fitted curve. Figures 8 and 9 show that the maximum cutting force and energy consumed by cutter *d* were higher than the other cutters. This is because cutter *d* has a small structure of the projecting tooth. The tip of the tooth of the cutter was able to easily stab the epidermis of the tea stalk but was very small, because of which more force was required to break the tissue structure of the tea stalk. These phenomena indicate that cutters *b* and *c* (biomimetic cutters) exhibited better cutting performance on the tea stalk than cutters *a* and *d*.

The article "Design of Structural Parameters of Cutters for Tea Harvest Based on Biomimetic Methodology" was published in 2021. Journal: Appl Bionics Biomech.

Cutters used to harvest tea plants are usually made of steel. However, to compare different cutters more accurately, this study used Future 8000 resin to manufacture them. In future work, the authors plan to make metal biomimetic cutters and measure their cutting forces and energy consumption. Further work in the area should also investigate the advantages of biomimetic cutters for different crops and at different loading speeds.

## 5. Conclusions

In this study, it was found that the cutting performance of cutters *b* and *c* was superior to that of cutter *a* at loading speeds of 5, 10, and 15 mm/s. Cutters *b* and *c* can use 9.43% and 6.04% less average maximum cutting force than cutter *a*, respectively, and required 13.8% and 4.24% less average energy at a loading speed of 15 mm/s. When the thickness of the cutter was 1.5~2 mm, the maximum equivalent stress and total deformation produced by cutters *b* and *c* did not change significantly. These results show that the first sharp tooth of the mandible of the cricket can be used to design biomimetic cutters that can cut the stalks of tea plants efficiently in terms of the cutting force and energy consumption.

## Figures and Tables

**Figure 1:** (a) Teeth on the mandible of the cricket. (b) Structure of the tea stalk.

**Figure 2:** Extracted contour line of the teeth of the cricket.

**Figure 3:** Best approximation of the fitted curve.

**Figure 4:** Best approximation of the fitted straight line: (a) rising portion and (b) falling portion.

**Figure 5:** Cutter models: (a) *a*, (b) *b*, (c) *c*, and (d) *d*.

**Figure 6:** Angles of the triangle.

**Figure 7:** Rule of equivalent stress and total deformation of the cutter with thickness.

**Figure 8:** Average maximum cutting force.

**Figure 9:** Average energy consumption at different loading speeds.

**Figure 10:** Structure of the tea stalk obtained through a micro-CT scanner. (a) Initial stalk. (b) Distorted stalk. (c) Damaged stalk.

**Figure 11:** Cutting force versus displacement.

**Table 1:** Parameters of the curve.

Parameters	Curve *a*	Curve *b*	Curve *c*	Curve *d*	Curve *e*
*a*_0_	3.248	–7.302	1283.896	41225.250	–16145.526
*a*_1_	5.295	1.689	–32.294	–420.6120	107.581
*a*_2_	0.104	–0.018	0.249	1.602	–0.263
*a*_3_	–0.006	7.08*e* − 05	–7.58*e* − 04	–2.70*e* − 03	2.83*e* − 04
*a*_4_	5.30*e* − 05	–1.04*e* − 07	8.00*e* − 07	1.69*e* − 06	–1.13*e* − 07
*R* ^2^	0.976	0.999	0.960	0.985	0.976

The article "Design of Structural Parameters of Cutters for Tea Harvest Based on Biomimetic Methodology" was published in 2021. Journal: Appl Bionics Biomech.

**Table 2:** Parameters of the fitted straight line.

Part	*b*_0_	*b*_1_	*R* ^2^
Rising portion	2.387	1.959	0.964
Falling portion	64.129	-1.891	0.953

**Table 3:** Maximum force during the cutting of the tea stalk.

No.	Loading speed (mm/s)	Maximum cutting force (N)			
		Cutter *a*	Cutter *b*	Cutter *c*	Cutter *d*
1	5	10.578	9.640	9.353	8.446
2		8.004	9.047	8.749	6.589
3		8.008	9.280	8.609	7.783
4		8.500	9.020	9.020	11.365
5		10.338	8.249	9.206	11.791

1	10	9.834	9.884	9.857	11.659
2		8.039	7.369	9.729	12.225
3		11.574	9.311	8.997	10.516
4		8.334	9.008	7.594	12.245
5		8.811	10.392	8.958	8.051

1	15	7.756	9.582	7.896	12.497
2		10.694	7.407	8.004	11.330
3		9.458	7.853	8.683	14.726
4		8.566	7.524	9.132	14.477
5		8.632	8.489	8.667	14.954

**Table 4:** Energy consumed to cut a single tea stalk.

No.	Loading speed (mm/s)	Energy consumption (J)			
		Cutter *a*	Cutter *b*	Cutter *c*	Cutter *d*
1	5	1.717	1.059	1.122	1.638
2		1.123	1.216	0.996	1.122
3		1.025	1.068	1.087	1.345
4		0.745	1.284	1.318	1.642
5		1.219	1.272	1.266	1.756

1	10	0.920	1.023	0.929	1.491
2		1.149	1.358	1.154	1.933
3		1.058	1.255	1.207	2.445
4		1.298	1.185	1.318	2.649
5		1.354	1.256	1.148	1.442

1	15	1.205	1.373	0.958	2.281
2		1.499	1.019	1.163	2.936
3		1.356	1.009	1.277	2.843
4		1.183	1.035	1.173	2.293
5		0.882	0.843	1.293	2.481

## Data Availability

The raw data used to support the findings of this study are included within the article.
